The article "Virulent Diuraphis noxia Aphids Over-Express Calcium Signaling Proteins to Overcome Defenses of Aphid-Resistant Wheat Plants" was retracted in 2017. Reasons: errors in the analysis; errors in the results or conclusions.

# Virulent *Diuraphis noxia* Aphids Over-Express Calcium Signaling Proteins to Overcome Defenses of Aphid-Resistant Wheat Plants

**DOI:** 10.1371/journal.pone.0146809

**Published:** 2016-01-27

**Authors:** Deepak K. Sinha, Predeesh Chandran, Alicia E. Timm, Lina Aguirre-Rojas, C. Michael Smith

**Affiliations:** 1 International Centre for Genetic Engineering and Biotechnology, New Delhi 110067, India; 2 Department of Entomology, Kansas State University, Manhattan, Kansas 66506–4004, United States of America; Huazhong University of Science & Technology(HUST), CHINA

## Abstract

The Russian wheat aphid, *Diuraphis noxia*, an invasive phytotoxic pest of wheat, *Triticum aestivum*, and barley, *Hordeum vulgare*, causes huge economic losses in Africa, South America, and North America. Most acceptable and ecologically beneficial aphid management strategies include selection and breeding of *D*. *noxia*-resistant varieties, and numerous *D*. *noxia* resistance genes have been identified in *T*. *aestivum* and *H*. *vulgare*. North American *D*. *noxia* biotype 1 is avirulent to *T*. *aestivum* varieties possessing *Dn4* or *Dn7* genes, while biotype 2 is virulent to *Dn4* and avirulent to *Dn7*. The current investigation utilized next-generation RNAseq technology to reveal that biotype 2 over expresses proteins involved in calcium signaling, which activates phosphoinositide (PI) metabolism. Calcium signaling proteins comprised 36% of all transcripts identified in the two *D*. *noxia* biotypes. Depending on plant resistance gene-aphid biotype interaction, additional transcript groups included those involved in tissue growth; defense and stress response; zinc ion and related cofactor binding; and apoptosis. Activation of enzymes involved in PI metabolism by *D*. *noxia* biotype 2 aphids allows depletion of plant calcium that normally blocks aphid feeding sites in phloem sieve elements and enables successful, continuous feeding on plants resistant to avirulent biotype 1. Inhibition of the key enzyme phospholipase C significantly reduced biotype 2 salivation into phloem and phloem sap ingestion.

## Introduction

Arthropods exhibit remarkable genetic plasticity in adapting to stresses posed by both abiotic and biotic factors. Among the arthropods, insect crop pests express virulence to virtually all insecticides and plant genes for insect resistance used for their control [1,2]. Presently, most insect species virulent to plant resistance genes are aphids (Homoptera) [3]. Virulence is presently identified by exposing an aphid population of unknown virulence capability to plant genotypes with different aphid resistance genes [4].

The molecular mechanisms of aphid virulence are poorly understood. The current state of knowledge suggests that when feeding, effectors in an avirulent aphid are recognized by the defense system of the resistant plant, the aphid cannot infest the plant. Conversely, when a normally resistant plant does not recognize aphid effectors, the virulent aphid overcomes the plant resistance gene or genes [5,6]. Evidence to date implicates the putative involvement of several aphid metabolic components of both salivary and gut origin in virulence [7–11].

Specialized aphid mouthparts consist of a tube-shaped arrangement of mandibles and maxillae that allow specialized stylet mouthparts to pierce plant tissues and create an extracellular pathway [12] to probe plant cells for nutrients. The fused maxillae form one tube for secretion of gelling saliva into plant tissues [13] and eventual secretion of watery saliva containing molecules that modulate plant cellular responses during phloem feeding [9, 14]. A second maxillary tube allows ingestion of preferred nutrients from phloem sieve elements. During compatible plant-aphid interactions, stylets reach the sieve elements and phloem sap is ingested [15], apparently due to the ability of aphid salivary proteins to bind plant calcium that normally occlude removal of phloem sap. In incompatible plant-aphid interactions, plant sieve element calcium occlusion allows only brief or no ingestion of phloem sap [16]. To date, the identity of aphid salivary proteins used to block plant Ca^2+^ influx remains unknown [17].

The Russian wheat aphid, *Diuraphis noxia*, (Kurdjumov) is a destructive global arthropod pest of wheat [18] that causes major wheat yield losses. Although numerous *D*. *noxia*-resistant varieties of wheat are deployed in North America and South Africa, the occurrence of *D*. *noxia* virulence to such genes continues [19–23]. *D*. *noxia* virulence is known to involve differences in aphid feeding behavior, growth and survival [24–26], but definitive results to demonstrate cause and effect relationships between molecular factors and virulence do not exist.

Given the compelling need to understand the molecular bases of aphid virulence, we explored the relationship between gene expression and virulence in *D*. *noxia* by comparing the RNAseq profiles of North American biotype 1 and biotype 2 aphids allowed to feed on wheat varieties containing no resistance, biotype 1 resistance or biotype 2 resistance. Our objectives were to: 1.) Identify biotype 2 virulence factors by comparing the transcriptomes of biotype 1 and biotype 2 feeding on plants containing the biotype 1-resistant, biotype 2- susceptible *Dn4* gene from wheat, *Triticum aestivum*; and 2.) Identify differences in avirulence and virulence biotype 2 proteins expressed in responses to *Dn4* plants to those from plants containing the *Dn7* gene from rye, *Secale cereale*.

## Results

### Transcriptome sequencing, assembly, and abundance estimation

The 18 *D*. *noxia* samples sequenced with the Hiseq 2500 sequencer generated 100 base pair single-end reads (see Materials and Methods). Each sample was represented by more than 20 million reads from each library, and >63.4% of the reads passed quality control (QC) “S1 Table”. The *Diuraphis noxia* genome sequence was unreported at the time of our experiments. Therefore, all reads that passed QC were pooled to generate a *de novo* assembly, which contained 253,744 contigs with N_50_ length of 1,855bp and a GC/AT ratio of 33.7/66.3% “S2 Table”. Reads from biotype 1 and 2 were then used to generate separate assemblies for each biotype. A total of 127,293 contigs with N_50_ length of 2,379 and 105,930 contigs with N_50_ length of 2,399 were generated for biotype 1 and biotype 2 samples, respectively. Read-contig alignments were performed to determine read support for transcript assemblies and to predict sample-wise utilization of reads. In each of the 18 aphid samples, reads passing QC were individually aligned to their respective assembly using pooled sequences. >91.5% of reads from each sample uniquely aligned to contigs generated using pooled sequences “S1 Table”. These results compare favorably with those in the *D*. *noxia* biotype 2 provisional genome [27], which contains 85,990 contigs (≥200bp) with N_50_ length of 2,863bp and GC/AT ratio of 32.8/67.2%.

### Differential expression analysis and functional annotations

RSEM (RNA-Seq by Expectation Maximization) software [28] was used in the *de novo* assembly to calculate RNA-seq reads derived from transcripts for downstream analysis. RSEM assigns reads to each transcript based on reads probability and generates transcript to gene maps using fasta files generated by Trinity. RSEM indicated that there was a greater abundance of transcripts than genes and multiple transcripts of the same gene, presumably resulting from alternate promoters, polyadenylation sites or alternate splicing. The analysis estimated 253,744 transcripts, >51,000 of which were expressed across all samples, and 204,094 genes, >42,000 of which were expressed across all samples.

Differential expression analysis by DeSeq software [29] revealed 26,373 transcripts and 20,804 genes in biotype 1 and 27,575 transcripts and 23,046 genes in biotype 2 commonly expressed among aphids feeding on the three wheat genotypes containing *Dn0*, *Dn4* or *Dn7* “Fig 1.” However, 197 transcripts and 178 genes were uniquely expressed in biotype 1 fed plants with no resistance genes (*Dn0)*, whereas 268 transcripts and 244 genes were unique to biotype 1 fed plants with the *Dn4* resistance gene, and 220 transcripts and 195 genes were unique to biotype 1 fed plants with the *Dn7* resistance genes. Biotype 2 fed plants with *Dn0*, *Dn4*, or *Dn7* uniquely expressed 146 transcripts and 137 genes, 206 transcripts and 189 genes, and 256 transcripts and 230 genes, respectively “Fig 1.” Numbers of significantly (>2 log_2_ fold) expressed transcripts and genes differentially expressed in each biotype in response to *Dn0*, *Dn4*, or *Dn7* are represented in Table 1.

**Fig 1:** Venn Diagram depicting total numbers of differentially expressed transcripts and genes in *D*. *noxia* fed wheat plants containing *Dn* genes for susceptibility (*Dn0* [brown circles]), biotype 1 resistance (*Dn4* [purple circles]) or biotype 2 resistance (*Dn7* [blue circles]). A (transcripts) and B (genes) in biotype 1, C (transcripts) and D (genes) in biotype 2.

**Table 1:** Numbers of significantly (>2 log_2_fold) expressed transcripts and genes in *D*. *noxia* biotypes 1 and 2 fed wheat plants containing the *Dn4* or *Dn7 D*. *noxia* resistant genes or plants with no resistance (*Dn0)*.

		Down-regulated		Up-regulated	
Biotype	R gene feeding comparison	Transcripts	Genes	Transcripts	Genes
1	*Dn0* versus *Dn4*	16	0	15	0
	*Dn0* versus *Dn7*	32	0	24	0
	*Dn4*versus *Dn7*	24	0	17	0
2	*Dn0* versus *Dn4*	11	0	9	0
	*Dn0* versus *Dn7*	18	1	18	0
	*Dn4*versus *Dn7*	21	3	36	8

DeSeq per-treatment comparisons yielded two-way contrasts of transcripts in *D*. *noxia* biotype 1 or 2 feeding on plants containing the *Dn0*, *Dn4* or *Dn7* plant genes in all possible combinations. In each treatment comparison, transcripts down-regulated in one treatment are up-biotype 2-susceptible *Dn4* compared to plants containing susceptible *Dn0* (no resistance) are shown in Table 2.

**Table 2:** Selected classes of transcripts from *D*. *noxia* biotypes 1 and 2 feeding on wheat plants containing the biotype 1 resistant-, biotype 2-susceptible *Dn4* gene compared to feeding on susceptible plants.

Responses of aviruelnt biotype 1			Responses of viruelnt biotype 2		
**Calcium signaling**					
**Comp ID**	Transcript ID *	**log 2 FC**	**Comp ID**	Transcript ID *	**log 2 FC**
39726c0seq15	elmo domain-containing 2 ^a^	5.8	40494c2seq4	PI-PLC X domain-containing	3.5
40953c0seq6	STK greatwall isoform	4.3	41519c0seq1	protein PFC0760c-like	3.5
36483c0seq5	PIGL	3.6	39271c0seq1	Niemann-Pick C1 protein	2.8
38315c0seq11	β-Ar3	3.2	34997c0seq6	synaptic vesicle glycoprotein	2.4
40352c1seq2	Ca+ channel subunit α2/δ3	2.3	39981c0seq17	rhogef domain-containing	−3.1
41703c0seq26	dynamin isoform X3	−3.6			
41451c0seq24	sterol regulatory element-binding/ cleavage protein	−3.1			
41359c0seq3	intersectin-1 isoform X2	−2.7			
38475c0seq5	clathrin light chain-like	−2.5			
**Stress response**					
20877c0seq2	aminopeptidase N-like	3.1	40354c0seq5	GABA Cl—channel subunit	−6.5
			41340c1seq11	LRR extensin-like	−5.5
			41311c0seq42	glucose dehydrogenase	−2.5
			38750c0seq2	trehalose transporter	−2.1
**Growth and development**					
41794c0seq1	C4b-binding protein β chain	3.1	41802c0seq16	homeobox protein cut i	4.3
40607c0seq28	PDZ/LIM domain Zasp ^b^	2.2	38574c0seq2	gastrula Zn finger protein	2.3
36581c0seq22	meiosis arrest female protein	−5.1			
36020c0seq2	helix-loop-helix protein 1	−2.9			
**Apopotosis**					
40719c0seq1	E3 ubiquitin ligase siah1	3.1			
39846c0seq1	tyrosine phosphatase ^c^	−2.4			
**Zinc and copper signaling**					
40324c0seq21	SOD copper chaperone	5.7			
40556c0seq44	Zn finger cchc/rna-bind motif	2.1			
40149c0seq19	E3 ubiquitin-protein ligase	−3.4			
41198c0seq2	Zn finger protein Xfin ^d^	−3.1			

* Unless noted, transcripts were similar to *A*. *pisum* sequences in BLASTX alignment; see “S3 Table” and “S4 Table” for complete transcript identifications.

^*a*^ *Zootermopsis nevadensis*

^*b*^ *Lygus hesperus*

^*c*^ *Anopheles darling*

^*d*^ *Apis mellifera*

Similar outputs for transcripts expressed in each biotype fed *Dn4* plants, plants containing biotype 1- and 2-resistant *Dn7*, and susceptible plants containing *Dn0* are shown in Table 3.

**Table 3:** Selected transcript classes in *D*. *noxia* biotype 2 feeding on wheat plants containing the *Dn4* gene from wheat, *Triticum aestivum*, or the biotype 2-resistant *Dn7* gene from rye, *Secale cereale*.

Responses to *Dn4*			Responses to *Dn7*			
**Calcium signaling**						
**Comp ID**	Transcript ID *	**log 2 FC**	**Comp ID**	Transcript ID *		**log 2 FC**
40494c2seq4	PI-PLC X domain-containing ^a^	3.5	41829c1seq19	rho guanine nucleotide exchange		3.8
41519c0seq1	protein PFC0760c-like	3.5	40856c0seq9	nuclear receptor coactivator		3.5
39271c0seq1	Niemann-Pick C1 protein	2.8	41260c0seq22	C2 transmembrane domain ^b^		3.2
34997c0seq6	synaptic vesicle glycoprotein	2.4	41503c0seq9	IQ motif/SEC7 domain ^c^		2.8
41415c0seq1	clathrin coat assembly protein **	4.6	41906c0seq40	trichohyalin isoform x1		2.6
35328c0seq2	ubiquitin-related modifier **	3.1	39849c0seq13	E3 ubiquitin ligase TRIM23 **		5.1
40836c1seq5	predicted tweety protein **	3.0	40494c2seq4	PI-PLC X domain-containing **		4.7
36982c0seq1	mitochondria Na+H+ exchange **	2.5	39573c0seq7	β l, 4 GalNAc bre-4-like **		3.0
37162c0seq3	lipase 3-like isoform X1 **	2.4	41640c0seq20	carnitine O-palmitoyltransferase **		2.6
37075c0seq2	O-GlcNAc transferase **	2.4	38475c0seq4	clathrin light chain isoform X3 ^d^ **		2.1
41421c1seq17	isoform I ^e^ **	2.2	37310c0seq3	multidrug R protein lethal		−3.5
39981c0seq17	rhogef domain-containing gxci	−3.1	40418c0seq3	CTP		−3.5
			40368c0seq9	tetratricopeptide repeat 8		−2.8
			39194c0seq26	E3 ubiquitin ligase TRIM33		−2.5
			41790c0seq11	calmodulin regulated spectrin		−2.5
			41706c1seq39	glucosylceramidase-like		−2.3
			36515c0seq4	DEF8		−2.1
**Stress response**						
39578c0seq1	cytochrome P450 CYP6CY3 ^f^ **	3.1	39509c0seq32		glucose dehydrogenase	5.2
41432c0seq7	carboxypeptidase d-like **	2.5	21361c0seq1		Hsp70-1 ^g^	4.1
41259c0seq9	mucin-17-like isoform X3 ^h^ **	2.2	39215c2seq1		autophagy related protein	3.8
38700c0seq1	cysteine protease ATG4B**	2.1	41432c0seq7		carboxypeptidase d-like	2.1
37605c0seq2	maltase A1 **	2.0	35396c0seq8		trehalose transporter **	2.4
40354c0seq5	GABA Cl—channel subunit	−6.5				
41340c1seq11	leucine-rich repeat extensin-like	−5.5				
41311c0seq42	glucose dehydrogenase	−2.5				
38750c0seq2	trehalose transporter	−2.1				

* Unless noted, transcripts were similar to *A*. *pisum* sequences in BLASTX alignment; see “S3 Table” and “S4 Table” for complete transcript identifications.

^a^ *Zootermopsis nevadensis*

^b^ *Zootermopsis nevadensis*

^c^ *Lygus hesperus*

^d^ *Apis mellifera*

^e^ *Pyrus x bretschneideri*

^f^ *Myzus persicae*

^g^ *Aphis glycines*

^h^ *Ctenocephalides felis*

** In DeSeq per treatment comparisons between responses to *Dn4* and *Dn7*, sequences up-regulated response to *Dn4* were down-regulated in response to *Dn7*. Sequences up-regulated in response to *Dn7* were down-regulated in response to *Dn4*.

Transcripts related to calcium-based signaling involved in PI metabolism constituted 36% of all transcripts identified. Virulence-based expression differences also occurred in tissue growth and development; stress response; zinc ion and copper signaling; and apoptosis (Tables 2 and 3).

Calcium signaling occurs when plasma membrane ion channels open after ligand binding of G protein-coupled receptors or receptor tyrosine kinases transduce extracellular signals across the cell membrane to mediate the activation of phospholipase C, a key element in PI metabolism “Fig 2” [30]. The major components of calcium signaling are rho GTPases that synergize signaling; receptor tyrosine kinase, which activates phosphatidyl-inositol 4,5 bisphospate (PIP_2_) a substrate for phosphatidylinositol 4,5-bisphosphate phosphodiesterase (PLC); PLC hydrolysis of PIP_2_ to produce inositol triphosphate (IP_3_); IP_3_-based release of Ca^2+^ from the endoplasmic reticulum; and diacylglycerol (DAG), which recruits protein kinase C and calcium ions. Protein kinase C (PKC) functions to desensitize G-protein receptors. β-arrestin (β-Ar3) is responsible for G protein uncoupling.

**Fig 2:** Calcium signaling in phosphoinositide metabolism. PIP_2_—phosphatidyl-inositol 4,5 bisphospate; PLC—phosphatidylinositol-4,5-bisphosphate phosphodiesterase-1; IP_3_—inositol triphosphate; DAG—diacylglycerol; PKC—protein kinase C.

### Biotype 2 virulence factors used to overcome *Dn4* in wheat

Quantitative and qualitative differences in the transcriptomes of biotype 1 and 2 ingesting phloem sap from *Dn4* plants provided several putative virulence factors in biotype 2. Avirulent biotype 1 up-regulated proteins to activate calcium signaling (elmo, PIGL, voltage-dependent calcium channel) but up-regulated STK greatwall to inhibit PLC and β-Ar3 “Fig 2” to quench calcium signaling and down-regulated dynamin, sterol regulatory, intersectin, and clathrin light chain calcium signaling proteins “Table 2”. In contrast, biotype 2 up-regulated PI-PLC (phosphoinositide-specific phospholipase C “Fig 2,” PFC0760c, Niemann-Pick, and synaptic vesicle proteins involved in calcium-based PI metabolism.

Biotype 2 also down-regulated a GABA transmembrane β chloride channel subunit (neurotransmission inhibition), and extensin- and trehalose transporter proteins involved in pathogen- and drought response, respectively “Table 2”. Biotype 1 up-regulated only an aminopeptidase N-like protein, a gut enzyme involved in arthropod virulence to endotoxins from *Bacillus thuringiensis*. Both biotypes up-regulated proteins involved in growth and development, but biotype 1 also down-regulated proteins involved in oogenesis (meiosis arrest female) and nervous system development (helix-loop-helix). Finally, biotype 1 also expressed proteins for apoptosis, and zinc and copper signaling. No such proteins were expressed in biotype 2 “Table 2”.

### Biotype 2 avirulence responses to the *Dn7* gene from rye

Differences in avirulence and virulence responses of biotype 2 were examined by contrasting the transcriptomes of biotype 2 fed plants containing *Dn4* from wheat to those of biotype 2 fed plants containing *Dn7* from rye. Biotype 2 produced over 50 transcripts of interest “Table 3”, and their expression differed considerably in response to plants containing either the *Dn4* or *Dn7* resistance genes. In *Dn4-Dn0* DeSeq comparisons, biotype 2 up-regulated four calcium-PI metabolism transcripts and down-regulated a rhogef domain-containing protein in response to *Dn4* “Table 3”. In the *Dn4-Dn7* DeSeq comparisons, biotype 2 up-regulated a unique collection of calcium homeostasis proteins only in response to *Dn4* (down-regulated in response to *Dn7*) “Table 3” and a unique group of defense proteins (carboxypeptidase d, cysteine protease, maltase, mucin, CYP6CY3) “Table 3”. As indicated in Table 2, biotype 2 down-regulated a GABA transmembrane β chloride channel subunit and extensin- and trehalose transporter stress response proteins.

More than twice as many calcium-PI metabolism transcripts were expressed by biotype 2 in response to *Dn7* plants than to *Dn4* plants, including those up-regulated with function as GTPases or in calcium binding in the absence of phospholipids, and several down-regulated proteins involved in lipid movement or PIP_2_ regeneration “Table 3”. A small collection of proteins was expressed only in response to *Dn7* (down-regulated in response to *Dn4*), including PI-PLC X, GTPase-activating E3 ubiquitin-protein ligase, carnitine O-palmitoyltransferase (lipid metabolism) and the clathrin light chain calcium ligand. Biotype 2 up-regulated only the carboxypeptidase d defense protein in response to *Dn7* and the Hsp70, Aut1- and FAD glucose dehydrogenase stress response proteins “Table 3”. Biotype 2 up-regulated a nearly equal number of growth and development proteins in response to both *Dn7* plants and *Dn4* plants “S2 Table” The most highly expressed were the PDZ/LIM domain (7.8-fold) and spectrin α chain (5.4-fold) muscle proteins in response to *Dn7* “S2 Table.” The midgut epithelial homeobox cut protein was expressed by biotype 2 in response to both *Dn4* (5-fold) and *Dn7* (4.3-fold) “S2 Table.” The PI-PLC X domain-containing protein, Tret1-like facilitated trehalose transporter, carboxypeptidase d and FAD quinone glucose dehydrogenase like proteins were expressed by biotype 2 in response to both *Dn4* and *Dn7* “Table 3”.

### REVIGO scatterplot analyses

Scatterplots of the most highly expressed transcript clusters in each biotype fed *Dn4* plants supported results in Table 2. Clusters up-regulated in biotype 1 fed *Dn4* plants “Fig 3A” represented increased transmembrane transport, signal transduction, and to a lesser extent, oxidoreductase activity, consistent with increased expression of calcium, copper and zinc signaling proteins “Table 2”. The most highly expressed clusters up-regulated by biotype 2 in response to *Dn4* plants also represented greater transmembrane transport, transferase-, catalytic, and lyase activity “Fig 3B”, consistent with up-regulation of PLC, PFC0760c, Niemann-Pick, and synaptic vesicle proteins involved in calcium-based PI metabolism “Table 2”.

**Fig 3:** Molecular functions of significantly expressed *D*. *noxia* transcript clusters up-regulated by biotype 1 (A) or 2 (B); and down-regulated by biotype 1 (C) or 2 (D) after ingesting phloem sap from wheat plants containing the biotype 1-resistant, biotype 2-susceptible *Dn4* gene compared to susceptible plants containing *Dn0*. Bubble color indicates p-value (legend in upper right-hand corner), bubble size indicates GO term frequency. See Methods Section for explanation of plot derivation.

After feeding on *Dn4* plants, biotype 1 down-regulated clusters for GTPase-, hydrolase and calcium binding activity “Fig 3C,” consistent with down-regulation of dynamin, intersectin, and clathrin light chain-like transcripts shown in Table 2. Down-regulated clusters in biotype 2 fed *Dn4* plants for diacylglycerol binding and GABA receptor activity, “Fig 3D” are consistent with down-regulation of a rhogef domain-containing protein, leucine-rich repeat serine/threonine-protein kinase, and GABA transmembrane β chloride channel subunit “Table 2”.

Clusters of transcripts produced by biotype 2 fed susceptible *Dn0* or *Dn4* plants or resistant *Dn7* plants differed considerably “Fig 4.” Those up-regulated in response to *Dn4* versus *Dn0 “*Fig 4A” are those shown previously in “Fig 3B” consistent with up-regulated calcium binding proteins in Tables 2 and 3. Clusters in “Fig 4B” representing transcripts up-regulated in response to *Dn4* but down-regulated in response to *Dn7* (as per this Deq per-treatment comparison) are shown in Table 3. A cluster expressed for protein transport represents up-regulated transcripts for clathrin coat assembly protein ap17-like and small ubiquitin-related modifier-like proteins involved in calcium re-absorption, homeostatis and transmembrane vesicular transport. A microtubule binding cluster represents up-regulated transcripts for protein tweety isoform and mitochondrial sodium hydrogen exchanger 9b2 isoform proteins involved in chloride and potassium movement across membranes to regulate cytoplasmic calcium. Monoxygenase, oxidoreductase and peptidase clusters represent CYP6CY3, maltase, cysteine protease, and carboxypeptidase. Clusters expressed for chitin binding and cuticle structure represent represent PDZ/LIM domain-, homeobox- and LOC100166146 proteins for muscle and epithelial tissue development “S2 Table.”

**Fig 4:** Molecular functions of significantly expressed *D*. *noxia* biotype 2 transcript clusters. (A) Clusters uniquely up- regulated in response to susceptible plants containing *Dn4;* (B) clusters up—regulated in response to *Dn4* plants but down-regulated in response to resistant plants containing *Dn7*; (C); clusters uniquely up- regulated in response to *Dn7* plants; (D) clusters up—regulated in response to *Dn7* plants but down-regulated in response to *Dn4* plants. Bubble color indicates p-value (legend in upper right-hand corner), bubble size indicates GO term frequency. See Methods Section for explanation of plot derivation.

Transcript clusters highly up-regulated by biotype 2 in response to *Dn7 “*Fig 4C” included a rho-guanyl-nucleotide exchange cluster representative of rho guanine nucleotide exchange factor 11, nuclear receptor coactivator 3 isoform x2 and IQ motif/SEC7 domain-containing protein 1; an O-acyl-transferase cluster representative of glucose dehydrogenase, heat shock and Aut1 stress response proteins; and a metallocarboxypeptidase cluster representative of carboxypeptidase d “Table 3”.

Major clusters for transcripts up-regulated in response to *Dn7* but down-regulated in response to *Dn4* (as per DeSeq per-treatment comparison) were transferase, transmembrane transport, ER signal peptide binding and signal recognition particle binding. The transferase cluster represented β-1,4 GalNac bre-4-like- and carnitine O-palmitoyl-transferase expression. The ER signal peptide-binding cluster represented clathrin light chain expression. A transmembrane transporter group represented trehalose transporter expression; and a signal recognition group represented expression of E3 ubiquitin-protein ligase TRIM23-like and PI-PLC X “Fig 4D”, “Table 3”.

### RT-qPCR

The over expression of biotype 2 transcripts capable of coding for proteins with substantial sequence similarity to several key enzymes involved in phosphoinositide (PI) metabolism led us to hypothesize about the involvement of the PI pathway in biotype 2-wheat interactions. When contigs with similarity to PLCγ1, DAG kinase, PKC, and β-Ar3 were subjected to RT-qPCR, PLCγ1, DAG kinase, and PKC in biotype 2 were 2^14^-, 2^6^-, and 2^3^-fold up-regulated, respectively, compared with expression of these genes in biotype 1 fed susceptible *Dn0* plants “Fig 5A, 5B and 5C.” A contig similar to a β-Ar3 was >2^10^-fold up-regulated in biotype 1 fed *Dn7* plants compared with biotype 2 fed *Dn7* plants “Fig 5D.” No amplification of PLCγ1 was observed in biotype 1 aphid fed *Dn4* plants, no amplification of β-Ar3 was observed in biotype 2 fed *Dn0* or *Dn4* plants. PLCγ1 primers amplified products only on biotype 2 template and β-Ar3 primers amplified only biotype 1 template (data not shown). PLCγ1 and β-Ar3 primers redesigned from a different location of each contig yielded similar amplification results. These results validate the over expression of PLCγ1 and β-Ar3 observed in biotypes 1 and 2, respectively, in the RNAseq expression analysis.

**Fig 5:** Relative expression (Mean ± SD) of (A) PLCγ1, (B) DAG kinase, (C) PKC, and (D) β-Ar3 in *D*. *noxia* biotype 1 and 2 aphids fed wheat plants containing the susceptible *Dn0* gene, the biotype 1 resistant, biotype 2 susceptible *Dn4* gene, or the biotype 1 and 2 resistant *Dn7* gene. Expression of PLCγ1, DAG kinase, and PKC calculated relative to expression of each gene in biotype 1 aphids fed *Dn0* plants. Expression of β-Ar3 calculated relative to expression in biotype 2 aphids fed *Dn7* plants. Asterisk (*) denotes no observed amplification.

### Aphid Feeding Bioassay

Mortality of biotype 2 after ingestion of the PLCγ1 inhibitor was assayed to determine the inhibitor concentration required to effect minimal changes in *D*. *noxia* feeding as measured by electrical penetration graph (EPG) analysis. The mortality of biotype 2 aphids fed artificial diet containing a 0.03mM concentration of the PLCγ1 inhibitor U-73122 increased from 10% mortality after 48h of feeding to 40% after 72h of feeding, compared to mortality on a control diet containing U-73343 (an inactive, non-inhibitory analog of U-73122) of 10% and 25% at 48- and 72h, respectively (data not shown).

### Aphid Electronic Penetration Graph (EPG) Analysis

EPG waveform analysis revealed that biotype 2 fed the U-73122 PLCγ1 inhibitor diet and then transferred to live plants containing the *Dn4* biotype 2 susceptible gene had significantly (*P <*0.05) more events of stylet penetration difficulty than biotype 2 fed control diet and required significantly (*P <*0.05) more cell punctures and intercellular probes during stylet salivation and tissue penetration than biotype 2 fed control diet “Table 4”. In addition, biotype 2 fed PLCγ1 inhibitor had significantly shorter periods of intercellular probing and completed significantly fewer cell punctures during the first intercellular probe than biotype 2 fed control diet.

**Table 4:** *D*. *noxia* biotype 2 feeding on *Dn4* wheat plants during an 8h EPG recording after 24 h of feeding on artificial diet containing either PLCγ1 inhibitor or control diet.

		Diet	
EPG Waveform	Mean (± SE) Feeding behavior	Inhibitor	Control
B—Stylet sheath salivation	Total cell punctures in 1st probe	1.8 ± 1.3 a	6.5 ± 1.8 b
	Total cell punctures	112.5 ± 14.2 a	48.3 ± 11.7 b
C—Intercellular stylet penetration	Number of probes	60.3 ± 8.5 a	22.6 ± 6.5b
	Duration of probing (min)	3.0 ± 0.1a	7.2 ± 0.1b
E1—Watery salivation into phloem	Median duration (min)	14.5 ± 5.9 a	59.9 ± 23.2 b
E2—Phloem sap ingestion	Median duration (min)	58.4 ± 24.5 a	225.1 ± 105.5 b
E1+E2—Phloem salivation & ingestion	Number of E1 + E2 events	25.0 ± 6.2 b	9.9 ± 2.6 a
	Duration of E1 + E2 events	117.5 ± 33.5 a	322.2 ± 102.7 b
F—Stylet penetration difficulty	Number of events	11.4 ± 1.4b	1.1± 1.1 a
G—Xylem sap drinking	Duration (min)	0.7 ± 0.03 a	6.6 ± 0.1b
	Number of events	14.1 ± 2.2b	6.0 ± 1.4 a

Within rows, treatment means followed by a different letter differ significantly (*P <* 0.05; Least Squares Means).

Biotype 2 fed PLCγ1 inhibitor diet exhibited significantly reduced median duration of watery salivation into phloem (EPG waveform E1), median duration of phloem sap ingestion (waveform E2) and mean duration of phloem ingestion and salivation than those fed control diet, but required significantly more salivation and ingestion events than those fed control diet (P<0.05) “Table 4”. In addition, biotype 2 fed PLCγ1 inhibitor diet also engaged in significantly more xylem sap drinking bouts than those fed control diet, and these were of significantly shorter duration than those fed control diet “Table 4”. These results demonstrate the inability of biotype 2 to deplete free extracellular phloem calcium during phloem feeding (cell punctures, E1, E2) and non-phloem feeding (stylet penetration, intercellular probes, xylem sap drinking) when the PLCγ1 enzyme controlling calcium signaling was inhibited.

## Discussion

Several key mediators in G-protein-coupled receptor (GPCR) reactions involve calcium signaling-mediated PI metabolism [31]. PIP_2_ regulates endoplasmic reticulum (ER) membrane dynamics and serves as a substrate for hydrolysis by PLC to generate IP_3_ and DAG [32], allowing IP_3_ binding with ER receptors, the release of ER calcium ions that bond with PKC [33], and stimulate uptake of extracellular calcium “Fig 2.” DAG kinase activation of PKC regulates phosphorylation and expression of several arthropod proteins involved in regulation of cold tolerance, diuresis, metamorphosis and salivation [34–37].

In avirulent responses to *Dn4*, *D*. *noxia* biotype 1 activates GPCR GTPases, yet simultaneously expresses STK greatwall protein to inactivate PLC activity, and β-Ar3, which curtails calcium signaling “Table 2”, “Fig 3”. The lack of PLC in biotype 1, along with the down-regulation of dynamin-, sterol regulatory-, intersectin-, and clathrin light chain calcium signals severely restricts calcium movement, resulting in avirulence [38]. Aminopeptidases, which exist in *D*. *noxia* saliva [9] have been suggested to function in *A*. *pisum* saliva in the detoxification of plant lectins [39]. An aminopeptidase N-like protein is 3.1-fold up-regulated in biotype 1 “Table 2”, but it appears to be ineffective in countering the defenses of *Dn4* plants.

Similar numbers of biotype 2 transcripts were expressed in response to plants containing *Dn4* from wheat or *Dn7* from rye, but the types of transcripts are quite different “Table 3”. Biotype 2 virulence to *Dn4* appears to be mediated by a combination of calcium signaling- and defense response factors “Table 2”, “Fig 3”. PI-PLC X, Niemann-Pick- and synaptic vesicle proteins interact to regulate calcium transmembrane lipid movement and generate DAG to remove calcium from *Dn4* plants. PLC is essential for larval and pupal development in *Helicoverpa armigera* [35], and increased PLC production in biotype 2 in response to *Dn4* may signal the increased production of homeobox- and gastrula zinc finger proteins “Table 2” to facilitate midgut epithelium repair, embryo development and increased biotype 2 survival.

Carboxypeptidase d, cysteine protease, maltase, mucin and CYP6CY3 “Table 3” all function in arthropod defense [40–43]. Ananthakrishnan et al. [7] have demonstrated production of trypsin-and chymotrypsin-like serine protease counter-defenses by biotype 2 to overcome *Dn4*. These results lend support to the hypothesis that after ingesting *Dn4* phloem, biotype 2 employs a suite of midgut defensive countermeasures to overcome resistance factors in *Dn4* plants. The down-regulation of the GABA transmembrane β chloride channel subunit, involved in neurotransmitter inhibition; and extensin- and trehalose transporter proteins involved in pathogen- and drought response “Table 3” adds additional evidence to suggest that biotype 2 relies primarily on calcium signaling- and midgut epithelium defenses to express virulence to *Dn4*.

Zn is essential for maintaining PKC structure and translocation through the plasma membrane [44,45]. Biotype 1 up-regulated both a CCHC type/RNA binding zinc finger protein and a SOD copper chaperone protein in response to *Dn4*, presumably to suppress ROS responses “S1 Table” but these were insufficient to overcome *Dn4* defenses. Biotype 2 expressed no Zn proteins in response to *Dn4*, but expressed a decaprenyl diphosphate synthase-like protein “S2 Table” responsible for synthesis of the ROS-related coenzyme Q_10_ antioxidant.

Biotype 2 produced more than twice as many calcium-PI metabolism transcripts in response to *Dn7* plants than to *Dn4* plants, including PI-PLC X and carboxypeptidase d produced to overcome *Dn4* defenses “Table 3”. However, biotype 2 down-regulated numerous proteins involved in calcium signaling, perhaps the most important of which are a differentially expressed in FDCP 8 homolog (DEF8) which contains a PKC conserved region with binding sites for DAG and RasGTPases; and phosphatidate cytidylyltransferase (CTP), required for PIP_2_ regeneration. Regardless of PI-PLC X expression, both DEF8 and CTP are necessary for the removal of free extracellular phloem calcium at aphid feeding sites. Biotype 2 also down-regulated glucosylceramidase-like-, multidrug resistance-, and tetratricopeptide repeat proteins involved in lipid metabolism; and an E3 ubiquitin-ligase trim 33 protein involved in calcium signaling. Finally, biotype 2 down-regulated calmodulin regulated spectrin-associated protein 1 (CAMSAP1), a nervous system microtubule-binding protein regulated by calcium-activated signaling [46]. The inability of biotype 2 to overcome *Dn7* defenses appears to be linked to the absence or reduced up-regulation of calcium signaling,- midgut defense response-, and ROS response suppression proteins used to overcome *Dn4*.

In contrast to biotype 2 fed control diet, biotype 2 fed PLCγ1 inhibitor and allowed to feed on plants containing the normally biotype 2-susceptible *Dn4* gene engaged in significantly reduced phloem feeding. Those fed control diet spent 67% of the 8 h EPG recording period (322 min) in phloem feeding compared to those fed inhibitor diet, which spent only 24% of the recording period (117 min) in phloem feeding “Table 4”. Biotype 2 fed PLC inhibitor for 24- to 72h also exhibited 2-fold down-regulation of PLC compared with those fed control diet (data not shown). Taken together, these results demonstrate the inability of biotype 2 to deplete free extracellular phloem calcium when PLC is inhibited and provide evidence to support our hypothesis that biotype 2 regulates plant calcium influx to prevent occlusion.

The osmotic effect of ingesting highly concentrated phloem sap provides an impetus for aphids to drink xylem sap, which is far less concentrated. Although biotype 2 fed PLC inhibitor diet engaged in significantly more xylem drinking bouts than those fed control diet, these were of significantly shorter duration than those fed control diet “Table 4”. These results further demonstrate the effects of PLC inhibition. Biotype 2 engaged in reduced phloem salivation and ingestion exhibited a corresponding reduced need to drink xylem sap.

Aphids encounter calcium in the plant epidermis, cortex and endodermis cells in route to the phloem, and the effects of PLCγ1 inhibition was present in the feeding behavior of *D*. *noxia* biotype 2 during encounters with these tissues as well. Biotype 2 fed PLCγ1 inhibitor exhibited significant increases in stylet penetration difficulties, plant cell punctures, intercellular probes, and ~10x greater incidence of derailed stylet activities compared to those fed control diet “Table 4”, suggesting that reduced calcium removal capacity adversely affects the feeding success of *D*. *noxia* when encountering calcium in these tissues.

The results of our experiments demonstrate differential regulation of PLC, PKC, DAG kinase, and β-Ar3 by *D*. *noxia* biotypes 1 and 2 in response to the phloem of plants containing the *D*. *noxia Dn4* and *Dn7* resistance genes. The over-expression of PLC, PKC and DAG kinase in virulent biotype 2 and the converse over-expression of β-Ar3 in biotype 1, each validated by RT-qPCR, clearly demonstrate the involvement of calcium signaling and PI hydrolysis in *D*. *noxia* virulence to *Dn4*. We hypothesize that *D*. *noxia* biotype 2 has evolved the ability to deplete free extracellular phloem calcium at numerous aphid feeding sites and feed on *Dn4* wheat plants normally resistant to avirulent biotype 1. Our results provide the first insights into transcriptome-based differences involved in *D*. *noxia* virulence and demonstrate the involvement of calcium-based PI metabolism and a suite of midgut defense- and insecticide resistance proteins in *D*. *noxia* biotype 2 virulence to overcome the *Dn4* aphid resistance gene in wheat. Future studies of PLC silencing or β-Ar3 over-expression will provide further insights into *D*. *noxia* virulence and avirulence.

## Materials and Methods

### Insect and plant material

*D*. *noxia* biotype 1 and biotype 2 aphids were collected from wheat fields near Hays, KS (38.8794° N, 99.3222° W), and Briggsdale, CO (40.6347° N, 104.3269° W), respectively, by employees of the USDA-ARS Plant Science Research Laboratory at Stillwater, OK. No specific permissions were required for these collections, as they were activities agreed upon by ARS scientists and scientists at Colorado State University and Kansas State University as a part of the Areawide Pest Management for Wheat: Management of Greenbug and Russian Wheat Aphid cooperative project between USDA-ARS and several states, including Colorado and Kansas. Field collections did not involve endangered or protected species. After collection, identity verification of each biotype was independently performed by plant differential diagnoses at Stillwater, OK, and Manhattan, KS. These aphids have been cultured in separate growth chambers in a Kansas State University greenhouse on susceptible wheat cultivar ‘Jagger.’ Specimen samples are also deposited at the Museum of Entomological and Prairie Arthropod Research at Kansas State University. Aphids of each biotype were starved for 12h before infestation of plants containing the biotype 1- and biotype 2 susceptible wheat variety Yuma, containing no resistance genes (*Dn0*); the biotype 1-resistant, biotype 2-susceptible wheat variety Yumar, containing the *Dn4* resistance gene; or the biotype 1, biotype 2-resistant wheat variety 94M370, containing the *Dn7* resistance gene [47]. Yumar is a near-isogenic line developed from a Yuma background containing *Dn4* [48]. The plants, potted in 16.5-cm-diameter-plastic pots containing Pro-Mix-Bx potting mix (Premier ProMix, Lansing, MI), were covered with fine screen mesh cages. Standard greenhouse conditions were maintained as determined previously [7, 49]. Apterous adult aphids were used for all the studies mentioned in this investigation. Post-infestation aphids were collected at 24, 48, 72 and 96h post-infestation and stored in RNAlater (Qiagen, GmbH, Hilden, Germany) according to the manufacturer’s recommendations.

### *D*. *noxia* RNA isolation, library preparation, and sequencing

Total RNA isolated from aphids collected at 24, 48, 72 and 96h post-infestation using the RNeasy Plus Kit (Qiagen, GmbH, Hilden, Germany) was quality-checked as mentioned in our earlier study [49], and equal amounts of total RNA (500ng) from each post-infestation time were pooled to form six treatments, including: biotype 1 fed plants containing *Dn0*, *Dn4* or *Dn7*, and biotype 2 fed plants containing *Dn0*, *Dn4*, or *Dn7* “S1 Fig”. 1μg of total RNA (100ng/μl) from each sample was used to prepare a TrueSeq library using an Illumina TrueSeq RNA sample preparation kit (Illumina Inc., San Diego, CA) per the manufacturer's recommendations. These libraries were validated, and a portion of each was diluted to a 10nM concentration. Samples were separately barcoded for multiplexing, and all libraries from 18 samples (6 treatments, 3 biological replicates) were combined into two pools (each loaded in 1 lane) of 9 libraries. A 1 x 100 bp single-read sequencing run was performed using an Illumina TrueSeq single-read clustering Kit v3 and Illumina TrueSeq SBS-HS v3 sequencing chemistry on an Hiseq 2500 Illumina sequencer. Library preparation and sequencing were conducted at the University of Kansas Medical Center in Kansas City, KS. Primary processing of sequences (conversion to FASTQ files, de-multiplexing) was completed at Genome International Corp. (Madison, WI). The sequence output, is available from the NCBI Short Read Archive (SRA) as SRA accession: SRP067435, effective March 31, 2016.

### Transcriptome assembly and abundance estimation

Before transcriptome assembly, PRINSEQ and FASTQC were used to remove adapter and low-quality sequences (Q ≤ 30) and duplicates. In the absence of a *D*. *noxia* genome sequence, 100 bp single base-pair high-quality reads from all 18 samples were used to construct a single *de novo assembly*, with Trinity assembling software [50]. k-mer size was fixed at 25bp. Similarly, separate assemblies for each biotype fed plants with different resistance genes were also generated to identify different alleles or unique genes. All short reads were assembled to form contigs without gaps, and reads from each sample were aligned back to assembled contigs separately. Only reads reported at least once in mapping were considered. Gene and transcript abundance were estimated using RSEM (RNA-Seq by Expectation Maximization) software for analysis of sequences generated from *de novo* assemblers of non-model species because it requires no sequence/genome information (http://deweylab.biostat.wisc.edu/rsem). RSEM estimates abundance of transcripts derived from a gene or isoform and the associated fraction of transcripts. Reads with ≥200 alignments were filtered out by RSEM maximum likelihood abundance estimates (transcripts per million), a fraction independent of mean expressed transcript length that includes a normalization factor. Following assembly with Trinity, TopHat was used to identify splice junctions. TopHat is a fast splice junction mapper for RNAseq reads that aligns RNAseq data using the ultrahigh-throughput short-read aligner Bowtie.

### Differential expression analysis

Transcripts from RNAseq data with a minimum relative log_2_ fold-change in expression and a threshold level of statistical significance (P_adj_ or q value < 0.1 to control false discovery rate) were selected to determine the significance of expression. All sequences were quality checked using OrthoDB (http://www.orthodb.org) to confirm transcript functional annotation. Those with conflicting results between BLASTX and OrthoDB were removed from consideration. The R/Bioconductor package DeSeq [29] was used to assess the statistical significance of differential expression. DeSeq uses a negative binomial distribution model to compare data in two groups to estimate the dispersion of differences between the groups to the variation within the group. The DeSeq per-condition (treatment) method was used to compare transcript expression using the three biological replicates in each of six treatments. The per-treatment comparisons determine that transcripts down-regulated in one treatment are up-regulated in the compared treatment and vice versa. Treatments included *D*. *noxia* biotype 1 or 2 feeding on plants containing the *Dn0*, *Dn4* or *Dn7* plant genes, with each of three treatment comparisons (*Dn4* to *Dn0*, *Dn7* to *Dn0*, or *Dn4* to *Dn7*) for each biotype.

BLASTX was used to find homologs of FASTA-formatted input sequences, which were aligned against NR, Swiss-Prot, and TrEMBL protein databases, using an E-value threshold of 0.001. Gene Ontology (GO) terms were assigned using BLAST2GO (http://www.blast2go.com/b2ghome). Differentially expressed GO terms from the UniProt database and p-values were included in the analysis. The REVIGO server (http://revigo.irb.hr/) was used to summarize GO terms and characterize differentially regulated contigs into large clusters, giving priority to enriched and statistically significant terms [51]. REVIGO scatterplot views were used to display representatives of significantly expressed transcript clusters after removal of redundancies in a two dimensional space derived from multidimensional scaling to a matrix of GO term semantic similarities. Sequences were annotated using Trinotate transcriptome functional annotation and analysis (http://trinotate.github.io*)* and homology searches of all known arthropod genomes.

### Quantitative Real-Time PCR

400ng of pooled total RNA was transcribed into first-strand cDNA using iScript RT Supermix (Bio-rad Laboratories, Hercules, CA) according to manufacturer’s recommendations. RT-qPCR primers for 20 selected genes were designed using Primer Express Software (Life Technologies, Grand Island, NY) “S5 Table”. RT-qPCR was performed on a CFX 96 Touch real-time PCR detection system (Bio-rad Laboratories, Hercules, CA). The RT-qPCR protocol was standardized according to MIQE guidelines, using previously determined detailed procedures [49]. 10 μl of RT-qPCR mastermix contained 1μl of synthesized cDNA, 1X iTaq Universal SYBR Green supermix (Bio-rad Laboratories, Hercules, CA), and 0.5 mM of forward and reverse primers. Fluorescence detection was performed at annealing temperature in all reactions, and cycling conditions were 95°C for 2 min followed by 40 cycles of 95°C for 30 s, 50°C or 60°C for 30 s, and 72°C for 30 s. Relative expression values were calculated based on the 2^−ΔCq^ method, a function of CFX Manager Software v3.0. Gene expression in biotype 1 fed Yuma (*Dn0*) plants was used as the calibrator. Actin and ribosomal protein L27 [49] were used as internal controls for all RT-qPCR assays. Melt curve analysis was performed for all reactions to identify primer dimers or contamination in PCRs. All PCR reactions were performed using three biological replicates and three technical replicates. Statistical software built into CFX Manager Software v3.0 was used to determine statistical differences between mean ± SD log_2_ fold-change gene expression.

### Aphid Feeding Bioassay

Experiments were conducted to inhibit PLCγ1 in *D*. *noxia* biotype 2 aphids fed U-73122, a PLCγ1 inhibitor [52,53] and a control diet containing an equal concentration of U-73343, an inactive (non-inhibitory) form of U-73122. The concentration of U-73122 causing minimal inhibition of aphid feeding was determined using serial dilutions from 0.17mM to 0.025mM final concentration in an artificial aphid diet developed by Febvay et al. [54] using 2mM stock. Aphids were fed a diet in parafilm sachets as described by Sadeghi et al. [55] with slight modifications. A thin sheet of sterile parafilm was stretched over the lid of a 50 x 9 mm Petri dish and 40 μl of diet solution was pipetted onto the parafilm. A second parafilm sheet was used to cover the medium on the first sheet. Ventilation was provided by small holes made with a needle in the Petri dish lid. Twenty mature biotype 2 aphids were then transferred into the Petri dish, and the cover containing the parafilm diet sachet was placed onto the dish. Aphids were counted after 24, 48, and 72h of feeding, and the U-73122 concentration at which 90% of aphids survived for 48h was determined and used to quantify changes in PLCγ1 expression (relative to aphids fed a control diet for 24h) and feeding behavior based on electrical penetration graph (EPG) analysis.

### Aphid Electronic Penetration Graph (EPG) Analysis

EPG experiments were carried out in the laboratory under continuous fluorescent illumination at 21–24°C and 40–45% RH. *D*. *noxia* biotype 2 aphids were fed an artificial diet containing U-73343 (control) or U-73122 (inhibitor) for 24h, starved for 4h in a Petri dish padded with sterile Whatman^®^No.1 filter paper. Each aphid was then tethered to a biotype 2-susceptible wheat plant containing the *Dn4* biotype 1 resistance gene by carefully attaching a thin (10–12 μm diam) gold wire (Johnson Matthey, Materials Tech, Royston, England) to the aphid dorsum using high-conductivity silver paint (SPI Supplies, West Chester, PA). The gold wire was soldered to copper wire and finally to a copper nail [56], which acted as the insect electrode. A copper wire inserted into the moist soil of each pot containing a plant with an aphid was the plant electrode [57]. Both electrodes were connected to a Giga-8 DC-EPG amplifier with 10^9^Ω input resistance and an adjustable plant voltage (Wageningen Agricultural University, Wageningen, The Netherlands) to record aphid feeding behavior. All plants were placed in a Faraday cage to decrease electrical noise. The output signal voltage was kept between +5 and -5 V. Care was taken to maintain the signal voltage as positive during the non-probing phase and as negative during intracellular punctures [13,57]. EPG output recordings were performed continuously for 8 h. EPG waveforms from 10 aphids (replications) fed either control or inhibitor diets were recorded using Stylet+ Software (EPG-Systems, Wageningen Agricultural University, Wageningen, The Netherlands). A built-in data logger (DI-710, Dataq Instruments Inc., Akron, OH) was used to digitize output recordings at 100 samples per sec.

*D*. *noxia* feeding behavior defined by established definitions [13,57] was measured for the number and duration of intercellular probes of the plant cell membrane by aphid stylets; the number of momentary intracellular punctures of the plant cell membrane; the number of stylet punctures in the first intercellular probe; the number of stylet penetration difficulty (derailed) events; the number and duration of watery salivation events into the phloem; the number and duration of phloem sap ingestion events; the number of xylem probes; and the duration of xylem sap drinking bouts. All EPG events were calculated using EPG-calc [58] and data were found to be non-normally distributed, according to the Shapiro-Wilk test of normality [59]. Waveform data were assessed to identify the transformation that most accurately explained the variance in the data. The gamma distribution, a two-parameter family of continuous probability distributions used for non-negative data modeling, was found to best explain treatment variances, as opposed to logarithmic or inverse square root transformations. The Satterthwaite method was used to estimate degrees of freedom [60] and the least squares means (P < 0.05) test was used for multiple comparisons of treatment means [61]. Transformed data were reconverted to the original scale for tabular presentation.

## Supporting Information

S1 Fig Experimental design for preparation of Illumina TrueSeq libraries of *D*. *noxia* biotypes 1 and 2 feeding on wheat genotypes and selection of genes for RT-qPCR. (PPT)

S1 Table Details of transcriptome sequencing, assembly, and transcript abundance for *D*. *noxia* biotypes 1 and 2 fed wheat plants with no resistance (*Dn0*) or plants containing the *Dn4* or *Dn7 D*. *noxia* resistance genes. (DOCX)

S2 Table Genome assembly statistics for *D*. *noxia* biotypes 1 and 2, as well as a pooled assembly. (DOCX)

S3 Table BLAST outputs and expression levels for significantly (>log2 fold) down-regulated and up-regulated transcripts in *D*. *noxia* biotype 1 fed plants containing different wheat *D*. *noxia* resistance genes. (XLS)

S4 Table BLAST outputs and expression levels for significantly (>log2 fold) down-regulated and up-regulated transcripts in *D*. *noxia* biotype 2 fed plants containing different wheat *D*. *noxia* resistance genes. (XLS)

S5 Table RT-qPCR primers designed from *D*. *noxia* genes used for gene expression studies in aphids feeding on different wheat genotypes. (DOC)
